# Long-Term Progression-Free Survival in a Patient with Locally Advanced, Unresectable Pancreatic Adenocarcinoma

**DOI:** 10.7759/cureus.406

**Published:** 2015-12-15

**Authors:** Brandon A Dyer, Leonel A Kahn, Mahan Matin, Richard J Bold, Michael I Tanaka, Arta M Monjazeb

**Affiliations:** 1 Radiation Oncology, UC Davis Medical Center; 2 Radiation Oncology, UC Davis Health System; 3 Pathology, UC Davis Health System; 4 Surgical Oncology, UC Davis Health System; 5 Hematology & Oncology, UC Davis Health System

**Keywords:** pancreatic cancer, chemotherapy, radiotherapy, surgically inoperable, progression-free survival

## Abstract

Pancreatic adenocarcinoma is amongst the most lethal malignancies with dismal five-year survival rates. Surgical excision is the mainstay of therapy and unresectable disease is considered incurable. Herein, we describe a patient with unresectable, advanced stage pancreatic adenocarcinoma with a remarkable clinical course following definitive chemoradiotherapy.

## Introduction

Pancreatic adenocarcinoma is amongst the most lethal malignancies with dismal five-year survival rates. Surgical excision is the mainstay of therapy, and unresectable disease is considered incurable. Unfortunately, early stage disease is often asymptomatic, and most patients are diagnosed with locally advanced or metastatic disease where surgical resection is not an option. Herein, we describe a patient with an unresectable, advanced stage pancreatic adenocarcinoma with a remarkable clinical course following chemoradiotherapy.

Written informed consent was obtained from the patient prior to drafting this text and no identifying information appears in this article.

## Case presentation

An otherwise healthy 69-year-old physician presented to his primary care physician for his annual physical with a three to four-month history of intense, episodic abdominal pain (8-10/10 in severity), which he attributed to a personal history of irritable bowel syndrome (IBS). He noted a 15-pound weight loss in the preceding several months and some fatigue but was otherwise without complaint. Aside from a family history of colon cancer in some distant relatives, his history was otherwise unremarkable with no history of alcohol, tobacco, or drug abuse. Informed patient consent was obtained prior to treatment.

Routine lab work during his annual physical revealed normal amylase levels and non-specific elevation of lipase (106U/L; 13-51U/L). His fasting blood glucose (BG) was also elevated at 145 mg/dL. Given the elevated BG, a basic metabolic panel was repeated several weeks later and was still elevated at 181 mg/dL.

Given the abdominal pain, elevated lipase, and new diagnosis of diabetes, the primary care physician ordered CT imaging to evaluate the abdomen and pelvis, which was completed six weeks after his initial presentation. CT imaging showed a 2.9 cm pancreatic mass encasing the celiac trunk and the proximal celiac arterial branches. Also noted were multiple, subcentimeter hypodensities throughout the pancreas with subcentimeter adjacent mesenteric lymph nodes, which demonstrated loss of fatty hilum, and were concerning for metastatic spread of disease (Figure 1).

**Figure 1:** CT scan of the abdomen and pelvis obtained at the time of diagnosis In the proximal pancreatic body, a poorly-defined hypodensity is seen with an apparent pancreatic duct cutoff sign (blue arrow), with pancreatic ductal distally. There is a relative loss of the normal fat planes surrounding the celiac artery as it branches into the splenic artery and common hepatic artery (red arrow). There are multiple, scattered shotty peripancreatic lymph nodes and an incidental peripheral hepatic hemangioma (yellow asterisk). The portal and hepatic vessels appear patent.

Subsequently, an endoscopic ultrasound with fine needle aspiration was performed, showing a highly cellular specimen containing clusters of malignant cells characterized by enlarged nuclei of different sizes and shapes with irregular nuclear contours and coarse chromatin. Some showed inconspicuous nucleoli. The cells also had a moderate amount of cytoplasm (Figures 2-3). A PET/CT scan demonstrated brisk FDG avidity of the pancreatic and peripancreatic tissue with subtle pleural-based left lung FDG avidity, which was felt to represent an inflammatory process. Carcinoembryonic antigen (CEA) was 1.9 ng/mL and cancer antigen 19-9 (CA 19-9) was 6.6 U/mL. He was evaluated by surgical oncology and deemed to be surgically inoperable with a clinical stage T4N1M0, Stage III pancreatic adenocarcinoma.

**Figure 2:** Hematoxylin and eosin stain of pancreatic fine needle aspiration Biopsy section at 10X magnification shows clusters of malignant cells forming acini. The cells have nuclei of different sizes and shapes with irregular nuclear contours and coarse chromatin.

**Figure 3:** Giemsa stain of pancreatic fine needle aspiration Biopsy smear at 20X magnification shows clusters of malignant cells with irregular nuclear contours and coarse chromatin.  Some show inconspicuous nucleoli. The cells also have a moderate amount of cytoplasm.

The patient was referred to medical oncology and was immediately started on systemic therapy consisting of folinic acid, 5-fluorouracil (5-FU), irinotecan, and oxaliplatin (FOLFIRINOX) and completed four cycles over the next two months. The patient tolerated chemotherapy with manageable adverse effects, including mild anorexia, nausea, fatigue, and overall malaise. The patient also noted improvement of his abdominal pain.

Repeat CT chest, abdomen, and pelvis obtained at the completion of FOLFIRINOX demonstrated stable proximal pancreatic hypodensities and unchanged encasement of the proximal celiac trunk and arterial branches, as well as stable peripancreatic nodes (Figure 4). Chest imaging showed no evidence of pulmonary metastases or lymphadenopathy.

**Figure 4:** CT scan of the abdomen and pelvis obtained after completion of FOLFIRINOX The distal pancreatic duct is dilated (blue arrow) and there is a poorly defined soft tissue mass at the pancreatic head and multiple hypodensities in the proximal pancreas, which encases the celiac axis (red arrow). There are multiple, scattered shotty peripancreatic lymph nodes and a stable, peripheral hepatic hemangioma (yellow asterisk). The portal and hepatic vessels appear patent.

The patient was subsequently referred to the Department of Radiation Oncology for consideration of radiation therapy (RT). At the time, the patient was asymptomatic and his physical examination was unremarkable. Laboratory data was notable for a fasting blood glucose of 156 mg/dL and normal ALT, AST, alkaline phosphatase, and total bilirubin. He had mild normocytic anemia (Hgb 12.5 g/dL, MCV 93μm^3^) and thrombocytopenia (104k/mm^3^) with other lab values within normal limits.

The patient was offered radiation therapy with a therapeutic goal of maintaining locoregional control and quality of life. Additionally, it was felt that a robust response could potentially make the patient a candidate for surgical resection. The patient was treated using intensity-modulated radiation therapy (IMRT) with an aggressive plan covering gross disease and suspicious lymph nodes with appropriate margins to 5400 cGy in 30 fractions and concurrent 5-FU by continuous infusion during radiotherapy. The patient completed radiation therapy nearly seven months after his initial presentation. The patient tolerated chemoradiotherapy with no major adverse effects. He did experience minor difficulty with nausea and “achy” abdominal pain, which resolved a few months after the completion of therapy. Subsequently, the patient elected not to receive further cycles of FOLFIRINOX due to moderate toxicity from the combined modality therapy.

The patient has received no further therapy since the completion of chemoradiotherapy as he was focused on quality of life and wanted to avoid a large, potentially non-therapeutic surgical procedure. CT imaging of the abdomen and pelvis obtained shortly after the completion of radiation showed an interval decrease in the size of the pancreatic mass (Figure 5). Serial CT imaging has demonstrated a continuous, progressive decrease in the size of the pancreatic and celiac axis mass. CEA and CA 19-9 laboratory values were followed and have remained relatively stable with time. 

**Figure 5:** CT scan of the abdomen and pelvis obtained after completion of RT There has been a drastic decrease in the mass and hypodensities in the pancreatic head (red arrow). The distal pancreatic duct is decompressed (blue arrow). There are multiple, scattered shotty peripancreatic lymph nodes and a stable, peripheral hepatic hemangioma (yellow asterisk). The portal and hepatic vessels appear patent.

MRI imaging obtained 33 months after his initial presentation and 26 months after the completion of radiation therapy demonstrated pancreatic atrophy with a residual fullness of the uncinate process. The celiac axis was widely patent with minimal surrounding ill-defined soft tissue. Additionally, there were preserved fat planes between the pancreas and the superior mesenteric artery and vein; otherwise, the imaging was unremarkable. On the most recent imaging, a CT scan that is more than 36 months after his initial presentation and 31 months after the completion of chemoradiotherapy, there is mild stable, ill-defined soft tissue fullness at the celiac axis, which likely represents post-treatment changes with no evidence of recurrent or progressive disease (Figure 6). The most recent CEA was 2.9 and CA 19-9 was less than 2.0 (lower limit of sensitivity for this assay). Clinically, the patient has been enjoying a remarkably excellent quality of life; six months ago, he had returned from a visit to see his grandchildren in Hawaii and was busy planning a river cruise in Budapest. The patient reports good appetite and energy level, regularly walking 8 miles daily with his dog. He experiences occasional abdominal discomfort, which he attributes to his IBS, but has no other complaints.

**Figure 6:** CT scan of the abdomen and pelvis obtained greater than 36 months after diagnosis There is pancreatic atrophy (blue arrow) with stable-appearing soft tissue surrounding the celiac axis (red arrow). There are stable-appearing peripancreatic lymph nodes and the previously seen peripheral hepatic hemangioma is no longer visible. The portal and hepatic vessels appear patent.

## Discussion

Herein, we have discussed the case of a patient with advanced pancreatic adenocarcinoma with a statistical life expectancy of 7.2 months who is now more than 36 months from his initial diagnosis with a durable clinical response and without evidence for recurrent or residual disease on serial imaging. Based on the American Joint Committee on Cancer, 7^th^ Ed., Stage III pancreatic adenocarcinoma corresponds to one, two, three, four, and five-year survival rates of 27%, 7.3%, 3.4%, 2.4%, and 1.8%, respectively, with a median survival of only 7.2 months [1]. Furthermore, there are very few reports of control of pancreatic adenocarcinoma and long-term progression-free survival without surgical intervention.

Pancreatic cancer has several known risk factors, which include tobacco use, diets high in animal fats, and exposure to noxious chemicals, including 2-naphthylamine, benzene, and gasoline. The most common presenting symptom is abdominal pain and jaundice secondary to common bile duct obstruction, which is indicative of high-grade, advanced disease on presentation.

Pancreatic cancer continues to be one of the most lethal malignancies, and there will be an estimated 48,960 new cases of pancreatic cancer in the United States in 2015, where pancreatic cancer is the fourth leading cause of cancer mortality in both men and women [2]. Worldwide, pancreatic carcinoma is the seventh leading cause of cancer mortality [3]. Unfortunately, despite advances in chemotherapeutic agents, targeted biologic therapies, immunomodulatory agents, and radiation therapy techniques, the trends in both disease incidence and overall survival have remained mostly unchanged and decidedly grim.

When feasible, the treatment of choice is surgical resection with pylorus-preserving pancreaticoduodenectomy used for lesions in the pancreatic head. With locally advanced, unresectable disease, the goal of therapy is to address the local disease burden, minimize locally obstructive symptoms, and convert to resectability, if feasible. There are several studies that established the role of chemoradiotherapy as a standard of care for locally advanced pancreatic cancer (LAPC), including the 1981 publication in Cancer by Moertel, et al. (GITSG-9273) and the 1988 Journal of National Cancer Institute publication by Douglas, et al. (GITSG-9283) that showed a statistically significant survival benefit with combined RT and 5-FU [4-5]. These early studies set the stage for subsequent trials evaluating various standard fractionation RT dose schema versus stereotactic body radiation therapy (SBRT) with neoadjuvant, concurrent, or adjuvant combinations of 5-FU, cisplatin, gemcitabine, capecitabine, erlotinib, irinotecan, and oxaliplatin [6-10]. Overall, the use of chemoradiotherapy versus chemotherapy alone in the definitive and adjuvant management of pancreatic cancer remains an area of controversy. 

This case proves that there may be a subset of patients for whom systemic disease control is possible and for whom local disease control can significantly impact clinical outcomes when treated with definitive chemoradiation. Considering the disease response in this patient and the paucity of clinical outcomes data in cases of pancreatic adenocarcinoma treated with definitive chemoradiation highlights the need for further clinical trials to identify patients who may benefit from definitive treatment and to better define the role of definitive radiotherapy.

## Conclusions

Despite continued research evaluating the etiology, timing, and molecular pathogenesis of pancreatic cancer, as well as new medical therapies, pancreatic cancer remains a common and deadly disease. Given the nearly universal, early mortality associated with the disease, the case presented herein is a remarkable example of disease response to definitive chemoradiotherapy and proves that definitive radiotherapy may play a role in a select subset of patients with pancreatic cancer.

## References

[1] (2010). AJCC Cancer Staging Manual, 7th Edition.

[2] American Cancer Society (2015). American Cancer Society Cancer Facts & Figures 2015. American Cancer Society.

[3] American Cancer Society (2012). American Cancer Society Global Cancer Facts & Figures 3rd Edition. American Cancer Society.

[4] Moertel CG, Frytak S, Hahn RG, O'Connell MJ, Reitemeier RJ, Rubin J, Schutt AJ, Weiland LH, Childs DS, Holbrook MA, Lavin PT, Livstone E, Spiro H, Knowlton A, Kalser M, Barkin J, Lessner H, Mann-Kaplan R, Ramming K, Douglas HO Jr, Thomas P, Nave H, Bateman J, Lokich J, Brooks J, Chaffey J, Corson JM, Zamcheck N, Novak JW (1981). Therapy of locally unresectable pancreatic carcinoma: a randomized comparison of high dose (6000 rads) radiation alone, moderate dose radiation (4000 rads + 5-fluorouracil), and high dose radiation + 5-fluorouracil: The Gastrointestinal Tumor Study Group. Cancer.

[5] The Gastrointestinal Tumor Study Group (1988). Treatment of locally unresectable carcinoma of the pancreas: comparison of combined-modality therapy (chemotherapy plus radiotherapy) to chemotherapy alone. J Natl Cancer Inst.

[6] Chauffert B, Mornex F, Bonnetain F, Rougier P, Mariette C, Bouché O, Bosset JF, Aparicio T, Mineur L, Azzedine A, Hammel P, Butel J, Stremsdoerfer N, Maingon P, Bedenne L (2008). Phase III trial comparing intensive induction chemoradiotherapy (60 Gy, infusional 5-FU and intermittent cisplatin) followed by maintenance gemcitabine with gemcitabine alone for locally advanced unresectable pancreatic cancer. Definitive results of the 2000-01 FFCD/SFRO study. Ann Oncol.

[7] Mukherjee S, Hurt CN, Bridgewater J, Falk S, Cummins S, Wasan H, Crosby T, Jephcott C, Roy R, Radhakrishna G, McDonald A, Ray R, Joseph G, Staffurth J, Abrams RA, Griffiths G, Maughan T (2013). Gemcitabine-based or capecitabine-based chemoradiotherapy for locally advanced pancreatic cancer (SCALOP): a multicentre, randomised, phase 2 trial. Lancet Oncol.

[8] Faris JE, Blaszkowsky LS, McDermott S, Guimaraes AR, Szymonifka J, Huynh MA, Ferrone CR, Wargo JA, Allen JN, Dias LE, Kwak EL, Lillemoe KD, Thayer SP, Murphy JE, Zhu AX, Sahani DV, Wo JY, Clark JW, Fernandez-del Castillo C, Ryan DP, Hong TS (2013). FOLFIRINOX in locally advanced pancreatic cancer: the Massachusetts General Hospital Cancer Center experience. Oncologist.

[9] Loehrer PJ Sr, Feng Y, Cardenes H, Wagner L, Brell JM, Cella D, Flynn P, Ramanathan RK, Crane CH, Alberts SR, Benson AB 3rd (2011). Gemcitabine alone versus gemcitabine plus radiotherapy in patients with locally advanced pancreatic cancer: an Eastern Cooperative Oncology Group trial. J Clin Oncol.

[10] Mahadevan A, Miksad R, Goldstein M, Sullivan R, Bullock A, Buchbinder E, Pleskow D, Sawhney M, Kent T, Vollmer C, Callery M (2011). Induction gemcitabine and stereotactic body radiotherapy for locally advanced nonmetastatic pancreas cancer. Int J Radiat Oncol Biol Phys.

